# Main Features of Business English Translation and Teaching Model Optimization Based on the Logistic Model

**DOI:** 10.1155/2022/2896349

**Published:** 2022-10-11

**Authors:** Jingying Huang

**Affiliations:** Recruitment and Employment Department, Sichuan University of Arts and Science, Dazhou, Sichuan 635000, China

## Abstract

With the continuous development of global trade in recent years, business English has received more and more attention as a medium of communication. Business English is a branch of English, and in order to meet the practical needs in business, business English is involved in various business disciplines from foreign trade to international logistics, to economics, foreign trade correspondence, law, and so on, which need to be translated in a more targeted manner. Therefore, there are many professional tutorials for business English in the market to guide trade personnel in business English translation. Many scholars have also conducted comprehensive studies on business English translation, some starting from its stylistic features and some focusing on translation skills, but fewer scholars have conducted studies on business English translation through models, and there is still a lack of theoretical basis for how to effectively improve the translation of business English. Therefore, in order to reduce the friction between different cultures in trade, promote business English better, and provide convenience for foreign traders, this study will implement the basic principles of “faithfulness, elegance” in English translation, with the aim of improving the practicality and effectiveness of business English, mainly from the main features of business English translation, and then, in the process of analysis, we mainly use the logistic model to analyze the characteristics of business English translation, including timeliness, professionalism, uniqueness, and diversity. The final analysis results show that the influence of professionalism and diversity on the effect of business English translation is more obvious, and we need to carry out a special teaching mode for these two points. The final analysis shows that professionalism and diversity have a significant impact on the effectiveness of business English translation, and special teaching models are needed to optimize these two points.

## 1. Introduction

The rapid development of business English is inseparable from the globalization of economy and trade. By the end of 2021, there are 73 countries in the world with nearly one billion people using English as their official language, and the importance of English is reflected by the number of countries, nearly 30% of which use English as their primary language. [1] Business English, on the other hand, is a business communication that aimed at adapting to the needs of the market, and it is a business that is specific to business services, forming business English which can penetrate into all aspects of business activities. With the development of the global trade industry, the role of English in the international arena is becoming more and more evident, and many industries are eager for business English translation professionals; so, more and more people are entering the industry. For these talents, business English is a necessary skill, which requires them not only to master professional English translation knowledge but also to understand the relevant processes of the foreign trade industry, understand the differences between different cultures, and understand how to deal with foreigners and talk business. Only in this way can the value of business English be put to good use and promote the continuous development of trade, which has also given rise to a series of teaching activities for business English, dedicated to better promote the development of business English. Based on this, in the modern society with continuous economic transformation and development, we should pay more attention to the relevant features and teaching modes of business English translation [2]. Among them, the number of English speakers and the number of international business English applicants are shown in Figure 1.

Translation of business English has certain characteristics. Unlike ordinary English, business English has its unique features in style, grammar, and syntax, which need more attention when translating. Some literature suggests that professional foundation is especially important for business English translation; some literature suggest that learning to be flexible and adaptable can accurately translate business English [3]. As can be seen, the findings of domestic and foreign scholars on this research topic are controversial. There are various characteristics of business English translation that have their own bases and have a certain influence on the accuracy and speed of translation, and the attention to any point in the translation process may affect the final result of translation [4]. Some scholars have found that business English is more specialized and some of the vocabulary come from the actual needs in the process of foreign trade. Moreover, the sentence style of business English is mainly for the purpose of understanding and requires more direct communication of information, so the sentence style is compact, logical, and has strong practicality. Gao Limin, a Chinese scholar, believes that linguistic features are very significant in the use of business English, which is more characteristic than the style of everyday English [5], and business English has its distinctive features in the expression of idioms and the transformation of specialized vocabulary [6]. However, there are few studies on the causal relationship between the effect of business English translation and its translation characteristics, among which there is a complex causal relationship between the effect of business English translation and the final translation results due to the large differences in the critique of the effect of business English translation and the lack of obvious embodiment of the characteristics, which makes it very difficult to identify the influence between the two [7]. An overview of the existing literature mostly explores the main features of business English translations from the aspects of comparison and examples, but there is less research on the inference of the degree of influence of these features, such as the study of the degree of influence of professionalism on the accuracy of business English translation results. It may be due to the fact that the most difficult problem to identify the influence of their features on conducting business English translation is the problem of model construction [8]. Therefore, the logistic model can be used as a tool to identify the effect of business English translation. The main differences between business English and ordinary English are shown in Figure 2.

This study uses SPSS 23.0 software to construct a logistic model for analysis. The contribution of this study is as follows: first, using the instrumental variable approach to solve the model construction problem, which makes the research results robust and error-free; second, analyzing the influence of business English translation features on its translation results is helpful to understand the influence of different features on translation effects [9]; third, to analyze the mechanism causes that affect the effectiveness of business English translation; fourth, it provides a reference for China to encourage and support the development of business English, improve the teaching level of related courses, and promote the continuous development of China's foreign trade in the context of economic globalization.

## 2. Research Background

There are many features of business English, and there is little literature to explore the research on the causal inference between the translation features of business English and the final translation results [10].

The literature review mainly revolves around the following parts: first, regarding the research on the translation characteristics of business English, foreign literature mostly adopts the methods of comparison and example to explore and analyze business English and everyday English. There are four main research results, which argue that the translation of business English has the characteristics of professionalism, timeliness, uniqueness, and diversity. Regarding the definition of professionalism, scholars generally believe that business English belongs to a branch of English, which has many fields, and some of them have special requirements and need to be translated according to the agreed rules in the industry in order to be better understood, such as shipping date, double check, B2B (Business to Business), C2B (Business to Business), and CBS (Business to Business). In addition, scholars also find that the translation of business English is very time-sensitive; because the international economic situation is changing rapidly, the translation of business English cannot be like the translation of ordinary foreign languages that have more ample time for revision and will lose its value in just a few days. Even some emergency messages can become useless in a few hours [11]. While information is changing rapidly, new technologies and products are emerging like a spring, and some relatively new products may not have professional terms to give their meanings, which requires business English to translate them as aptly as possible in the process of translation, showing the uniqueness of business English at the forefront of economic trade and providing reference for subsequent translators. The last is that in business English, a branch of English, many tenses and grammars are executed according to the English standard but need to be combined with the latest laws and regulations and proper nouns, so that business English will be flexible in the process of translation according to the actual situation to better meet the understanding needs of readers and fully reflect its diversity [12]. The main features of business English translation as currently considered by the mainstream are shown in Figure 3.

Second, the research on business English teaching strategies is considered. According to the research of foreign scholars, business English has its special linguistic characteristics, and in the process of trade, different translation needs will arise due to different cultures, which requires targeted teaching and counseling in the process of teaching these characteristics. Therefore, first of all, teachers need to have solid business English translation skills, be able to translate according to certain translation rules, and to summarize these translation strategies. In contrast, Wei Hua, a domestic scholar, discussed the feasibility of targeted teaching in terms of theoretical foundation and practical application of business English from the background of education informatization and verified the effectiveness of the new teaching model in three following aspects: improving students' business English foundation, improving teachers' business English teaching ability, and updating the teaching mode.

Third, scholars' different choices in the selection and use of research methods and research theories of the two can cause certain bias in the research results. In the process of analyzing the characteristics, scholars mostly use simple research methods such as illustration and comparison highlighting; this descriptive analysis is easy, but the analysis perspective is single and limited, and it may not be possible to present the correct and unmistakable result analysis in the complex cause-effect relationship. One of the most important problems faced by choosing a model for inferential analysis is that the model itself has the problem of endogeneity, and if it is not solved, then the inferred results will also be biased [13]. Some other scholars have inferred the relationship between the two through qualitative studies, and this approach has some limitations. In terms of research on the teaching model, most scholars use the 4ES criteria and believe that when translating business English, the effectiveness of translation will be considered in terms of its characteristics, for example, in order to better achieve accurate business English translation, i.e., to accurately complete the communication and delivery of information between different traders, teachers are required to pay attention to the professional basis of explanation [14]. By comparing the characteristics of professionalism, abbreviation, and rhetoric in business English vocabulary, foreign scholars require the popularization of these characteristics in teaching in order to improve the final translation skills [15].

To sum up, the analysis of the features and strategies of business English translation in China still remains in the comparative analysis of theories and examples, and the method of causal inference between various features has not been fully applied to this field. Therefore, this study will make up for the deficiencies of the previous studies by analyzing and studying the features and mechanisms of business English translation, which will help explore the influence of various features on the effect of business English translation and actively improve business English. It will help to explore the influence of various features on the effectiveness of business English translation and actively improve the relevance of business English teaching.

## 3. Materials and Methods

### 3.1. Basic Theory

#### 3.1.1. The Logistic Regression Model

The logistic regression model generally belongs to the dichotomous dependent variable model, that is, the dependent variable (generally *y*) in the model will be divided into two complementary results for analysis, such as whether it travels and whether the results are reasonable, which is more common in academic research. Its uniqueness lies mainly in its method of parameter treatment; generally, we use linear regression in linear equations, while logistic uses the maximum likelihood estimation method [16]. In the process of data analysis, the maximum likelihood values will have the characteristics of consistency, asymptotics, and asymptotic normality [17]. The business English translation effect of the respondents of this study is expressed by *Y* under the action of independent variables of several groups of characteristics, and its assignment rule is as follows: 1 = good translation effect and 0 = bad translation effect. Let the probability of the good translation effect be P and the probability of the bad translation effect be *Q*. *x*1, *x*2, *x*3, and *x*4 denote the four factors that affect the result *Y*. The evaluation criteria of the four factors are indicated by 1 for satisfied and 0 for unsatisfied, as shown in Figure 4.

#### 3.1.2. The Main Evaluation Method

In this study, we established a logistic regression equation to analyze the translation of business English in real life. However, we cannot analyze and predict the equation directly. In order to more accurately reflect the relationship between the independent and dependent variables, statistical methods are also needed to conduct tests, which are commonly used, namely, the value of the statistic of the regression coefficient test and the standard deviation of the estimated quantity, generally expressed by Wald and S.E. In addition, the Wald test will take into account its probability of significance (Sig), which will be compared by exp (*β*) [18].

(1) $$\begin{array}{c} S.E.=\sqrt{var\left(\beta \right),} \end{array}$$

(2) $$\begin{array}{c} Wald=\frac{\beta^{2}}{var\left(\beta \right)}\text{.} \end{array}$$

Generally, we will use 1% or 5% as the test threshold for the significance level, on the basis of which the corresponding value is tested, and less than or equal to the result is considered significant. And some models will use a more precise Sig value to determine the significance. Assuming the premise that the regression coefficient is equal to 0, followed by the calculation of the Sig value, the implication is that the probability that the coefficient estimated by the model will not be smaller than the known coefficient [19]. After calculating the results, even if the original hypothesis has been established, it is still necessary to test whether the Sig value is as expected, and generally, the smaller the Sig value, the less likely the hypothesis will be valid and vice versa, which means that the original hypothesis is valid. Generally, we use SPSS, Excel, and other calculation software to obtain the Sig value [20]. In (1), the size of S.E. reflects the degree of fluctuation of the estimator in the process of taking values, and when the smaller the S.E. is, i.e., the larger the Wald, the higher the importance of the independent variable in the regression equation.

In addition to this, in the regression equation, a one-sample *t*-test is also conducted to analyze whether there is a significant difference between the mean value of a variable and the specified test value; generally, the null hypothesis for a one-sample *t*-test is expressed as H0; there is no difference between the mean value and the specified test value. After that, the significance level is compared with the Sig value, which is less than or equal to reject H0, and the opposite is accepted.

Finally, after standardized analysis of the equation, all the relationships between the independent and dependent variables are measured in the same units; although their units may be different in the process of actual measurement, they are also more comparable after substitution into the equation.

### 3.2. Model Setting and Variable Selection

In order to solve the endogeneity problem in the above study and to perform unbiased estimation, the instrumental variables are chosen to solve the endogeneity problem. Because of the unique advantages of the instrumental variables approach used in this study, compared to the limitations of other research methods, the data in this study have exceptionally good statistical significance.

#### 3.2.1. Model Setting

A model of business English translation effectiveness is first established with the following equations:

(3) $$\begin{array}{c} P=\frac{\left(e^{{\;\beta }_{0}+\beta_{1}X_{1}+\beta_{2}X_{2}+\beta_{3}X_{3}+\beta_{4}X_{4}\;}\right)\;}{1+e^{{\;\beta }_{0}+\beta_{1}X_{1}+\beta_{2}X_{2}+\beta_{3}X_{3}+\beta_{4}X_{4}\;}}\text{,} \end{array}$$

where *P* denotes the probability of a good business English translation result. *X*_*i*_ is a series of variables, such as timeliness, professionalism, uniqueness, and diversity. Since *P* + *Q* = 1, the equation for the probability of a bad business English translation result can be obtained according to the following equation:

(4) $$\begin{array}{c} Q=\frac{1\;}{1+e^{{\;\beta }_{0}+\beta_{1}X_{1}+\beta_{2}X_{2}+\beta_{3}X_{3}+\beta_{4}X_{4}\;}}\text{.} \end{array}$$

From (4), it can be seen that there is a curvilinear relationship between the effect of business English translation and the variables of interest, and the ratio between the two formulas *P* and *Q* is defined as the occurrence ratio odds.

(5) $$\begin{array}{c} O\;d\;d\;s=\frac{P}{Q}e^{{\;\beta }_{0}+\beta_{1}X_{1}+\beta_{2}X_{2}+\beta_{3}X_{3}+\beta_{4}X_{4}\;}e^{{\;\beta }_{0}\;}e^{\beta_{1}X_{1}\;}e^{\beta_{2}X_{2}\;}e^{\beta_{3}X_{3}\;}∙e^{\beta_{4}X_{4}}\text{.} \end{array}$$

Taking the natural logarithm, there are

(6) $$\begin{array}{c} \text{Ln}=\frac{P}{Q}{\;\beta }_{0}+\beta_{1}X_{1}+\beta_{2}X_{2}+\beta_{3}X_{3}+\beta_{4}X_{4}\text{.} \end{array}$$

In this equation, *β*_0_, *β*_1_, *β*_2_, *β*_3_, and *β*_4_ are the relevant regression coefficients, where (4) is a nonlinear equation, which is commonly solved by the Newton–Raphson method.

#### 3.2.2. Data Sources

The data used in this study are all survey data, collected through the online release of questionnaires and used for analysis after collation. In the course of the survey, 285 valid questionnaires were obtained.

The number of business English users accounted for 51.25% of the total sample; among the respondents' education, 82.58% of the total sample was bachelor's degree or above, and 75.82% of the total sample aged between 22 and 25. Through the above statistical analysis of the sample, it is clear that most of the respondents are young people in their 20s, with higher education level, and they have a better understanding of the questionnaire content; so, the data of this research activity have high reliability and representativeness. Using SPSS 23.0 software for reliability analysis, the survey used the Cronbach coefficient, which was calculated as 0.815, the best reliability coefficient, indicating that the questionnaire was designed reasonably. In addition, the sample adequacy was assessed by the KMO coefficient, and the calculated result was 0.889, which is a high level, indicating that the number of samples in this survey meets the requirements and the adequacy is good. Finally, the distribution of the data was also analyzed, and the Bartlett value was chosen to measure it, with a value of 1527.942. After performing the calculation, the test value obtained was 0.01, which is less than the hypothesis of 0.05, indicating that the distribution of the survey data obtained is more reasonable.

#### 3.2.3. Definition of Variables and Descriptive Statistics

Dependent variables: timeliness of business English translation, professionalism of business English translation, uniqueness of business English translation, and diversity of business English translation are the dependent variables. This study focuses on the effects of these four characteristics on the effectiveness of business English translation. This study uses a variety of combined data to measure this indicator of the effectiveness of business English translation. The answers to the questions in the original questionnaire are divided into four categories, and this paper re-establishes a dichotomous variable as the dependent variable through the above questions and answers. Any translation result that gets a rating greater than or equal to 75 is recorded as 1, regardless of the specific value; any rating less than 75 is always recorded as 0, indicating a bad translation effect.

Independent variable: the translation effect of business English is the independent variable. In this study, the translation effect of business English is reassigned as a dichotomous variable, and the selected item is assigned a value of 0 for the good translation effect, while the rest of the variables are set as the bad translation effect and assigned a value of 1.

Control variables: English usage, English grammar, and users' English level are the control variables. There are many factors affecting the effect of features on the business English translation effect, which must be controlled in the model as much as possible, and the control variables in this study include three categories.

This work studies the effect of business English translation features on translation results, so the questions used are sample sizes selected from business English exams. Most of the question topics are from the International Business English Qualifying Examination, and a small number of topics are from other teaching and learning materials.

English usage variables including business English, test-taking English, and everyday speaking are not normally distributed.

English grammar variables including whether there are grammatical errors, correct tenses, and spelling errors are generally assigned as dichotomous variables.

User's English level variables including respondents' English level and frequency of exposure to English are generally classified as unfamiliar, beginner's level, mastery level, and proficient level-by-level, and here, the default respondents are all at mastery level to better analyze the influence of translation characteristics on their results. The distribution of respondents' English levels is shown in Figure 5.

## 4. Results and Discussion

### 4.1. Analysis of Descriptive Statistical Results

In this survey on the translation characteristics of business English, it involves timeliness, professionalism, uniqueness, and diversity. For better statistical analysis, the questions released will be classified according to these four characteristics, and after the respondents answer the questionnaire, they will then be divided into two following kinds in total: the questionnaire with a good translation effect and the questionnaire with a bad translation effect. These four characteristics are divided into three levels: 0 = no significant characteristics, 1 = average characteristics, and 2 = significant characteristics. First, the statistical results of the questionnaire with a good translation effect are analyzed, as shown in Figure 6.

Next is the analysis of the statistical results of the questionnaire with the poor translation effect, as shown in Figure 7.

This time, the total characteristics of all questionnaires were statistically analyzed, as shown in Figure 8.

In the description of the model variables in this study, first, the explanatory variable is the categorical variable of good and bad business English translation effects, which represents “whether the translation score meets the requirements in the completed business English test,” 0 = bad translation effect, and 1 = good translation effect. The next is the explanatory variable, and the four features selected in this study are all categorical variables: (1) timeliness, 0 = features not significant, 1 = features average, 2 = features significant; (2) professionalism, 0 = features not significant, 1 = features average, 2 = features significant; (3) uniqueness, 0 = features not significant, 1 = features average, 2 = features significant; (4) diversity, 0 = features not significant, 1 = features average, 2 = significant.

### 4.2. The Variable Correlation Test

Among the many methods for identifying causality, SPSS has a more obvious advantage for the comparison between variables. So, in this study, SPSS software is selected for calculation to solve the correlation problem of the model, and the correlation results are given in Table 1.

Among the four translation characteristics of business English, there is a positive correlation between timeliness and the explanatory variables, which indicates that more timeliness for business English will get a better translation effect, which is more in line with the actual needs in trade. Similarly, there is a positive relationship between professionalism, diversity, and the explanatory variables, indicating that the significance of these two characteristics plays a positive role in how well business English is translated. On the other hand, uniqueness is negatively correlated with the explanatory variables, indicating that this feature does not have a positive effect on the translation effectiveness of business English. This is consistent with what was expected at the beginning. In addition, there are positive and negative relationships between different variables, which are consistent with the basic rules of the model, for example, the negative relationship between uniqueness and diversity and the positive relationship between uniqueness and professionalism, which is basically in line with common sense. From the overall data of the table, the absolute values of the correlation coefficients between all variables are less than 0.5, and there is no excessive situation, which is within a reasonable range. It shows that the correlation between these four characteristics is weak, and the variables are more independent from each other, which meets the requirements of the setting of compound variables, and the preliminary judgment is that there is no colinearity between the variables, and the next step of analysis can be conducted.

### 4.3. Estimation Results of the Logistic Model

The statistical results in this study have good statistical significance, including ^*∗∗∗*^*P* < 0.01, ^*∗∗*^*P* < 0.05, and ^*∗*^*P* < 0.1. Considering the complexity of the operation, the data with 95% confidence interval is selected as the result in this study. According to the above model and related data, after the iterative operation, the final distribution parameters of the logistic probability model are *β*_0_ = 0.062, *β*_1_ = 0.067, *β*_2_ = 1.824, *β*_3_ = 0.526, and *β*4 = 1.241, so the final derived business English logistic probability distribution function of the effect of translation features on the translation effect is as follows:

(7) $$\begin{array}{c} P=\frac{\left(e^{0.062+0.067X_{1}+1.824X_{2}+0.526X_{3}+1.241X_{4}\;}\right)\;}{1+e^{0.062+0.067X_{1}+1.824X_{2}+0.526X_{3}+1.241X_{4}}}\text{,} \end{array}$$

where Sig *f* = 0.001, which is less than 0.005, indicating that it passes the validity test within the 95% confidence interval and the statistical results are reliable.

### 4.4. Analysis of the Mechanism by Which the Main Features of Business English Affect Its Translation Results

This study analyzes four characteristics of business English translation and the first of all is the timeliness of business English. The regression coefficient of the translation effect affected by the timeliness of business English is 0.067 (*t* = 2.24, *P*=0.005 < 0.01), which is significant at the 5% level, indicating that timeliness has a significant positive effect on the translation effect of business English. It can be said that the stronger the timeliness of English, the better its translation effect and the easier it is to accurately use English to convey information among people of different cultures, especially in the more pragmatic import and export trade, where the timeliness of business English is regarded as very important, and the communication by phone, fax, or e-mail in a short period of time can greatly affect the final translation effect because of the timeliness, which is consistent with the previous expectation.

The second is the professionalism of business English; generally, some fixed words or phrases are used in business English, which are required to be standardized and specialized in certain processes, and are bound by some official documents or rules. In the logistic model of this study, the final estimation result shows that the regression coefficient of professionalism in business English is 1.824 (*t* = 1.526, *P*=0.000 < 0.01), which is significant at the 5% level, indicating that professionalism has a positive impact on the final translation of business English. In the process of translation, we can better translate the meaning of both parties, use short words or sentences that are easy to understand but professional, and improve the translation effect.

Next is the uniqueness of business English; some common English words will be given special meanings in business English, which can be applied in the original context and adapted to the new business English environment, reflecting a good translation effect. Of course, this is based on the premise that the business English level of the users is still good, which is more conducive to the translation effect of business English. In the logistic equation of this study, the coefficient of business English uniqueness is 0.526 (*t* = 4.126, *P*=0.01 = 0.01), which seems to have a positive effect on the translation of business English, but the *P* value of its test is 0.01, which means that this result is not very significant and does not fully pass the 5% significance test. Combined with the previous respondents' English proficiency, the preliminary analysis is due to the different business English proficiency of the respondents and more deviations in the understanding of particular words.

Finally, the coefficient *X*3 of diversity of business English is 1.241 (*t* = 3.51, *P*=0.001 < 0.01) from the results of regression analysis, which is significant at the 5% level, indicating that the diversity of business English has a significant positive effect on its translation effect, and the more diverse the meanings of words, the more important they are in the process of translation and the more prominent they are for the overall translation effect. The more diverse the meanings of the words, the more important they are in the translation process and the more prominent they are for the overall translation effect. This indicates that significant diversity in business English can significantly improve the translation effect of business English.

On the whole, the timeliness, professionalism, and diversity of business English have a significant impact on its translation effect. Especially, professionalism and diversity have a greater impact on achieving good translation effects.

## 5. Conclusion

This work mainly studies and analyzes the translation characteristics and translation effects of business English, so as to obtain relevant suggestions for the optimization of the teaching mode and solves the correlation problem among variables by SPSS software calculation, so as to achieve the maximum likelihood estimation. The results of the estimation show that, first, the timeliness, professionalism, and diversity of business English translation have an impact on the translation effectiveness of business English. Second, further studies on the influence mechanism show that the professionalism and diversity of business English have more significant effects on the translation effectiveness of business English.

Business English is a professional English and a cross-disciplinary discipline, and its translation is different from traditional British or American English, which only requires learning the corresponding grammar knowledge and mastering a certain amount of vocabulary to complete the translation and achieve better results. In business English, however, due to its timeliness, professionalism, uniqueness, diversity, or other characteristics, translators are significantly affected by these characteristics in the process of translation and need to pay attention to the multiple meanings of words and the timeliness of translation through their accumulated professional knowledge in order to achieve better translation results. In this context, many experts and scholars study about the mode of teaching business English and analyze how to better optimize the existing business English teaching. In summary, based on the results of previous model analysis and mechanism research, this study comes up with the following suggestions for optimizing the business English teaching model.

- Choose accurate word meanings: In business English, the same word is likely to have multiple meanings, a phenomenon often encountered in the learning process of general English and even more so in business English, where many words have multiple meanings and are applicable to different contexts. Generally, such words with multiple meanings, such as literal, derived, extended, connotative, and extended meanings, need extra attention in the translation process. Therefore, teachers need to clarify this point when instructing business English translators, remind students of the concept of multiple meanings of words, and strengthen their awareness in this area through repeated practice of typical topics. For example, the most common literal meaning of the word “accident” is “accident,” but there are also other meanings such as “traffic accident, accidental event, unpredictable event.” Take out accident insurance before you go on your trip. The word “accident” is more in line with the context because there is an “insurance” with it, but if translated as other meanings, it is not very reasonable here. Another example is that talking to others can often help to put your own problems into perspective. In this sentence, the common meaning of “perspective” is “attitude, point of view,” which is used as a noun. But considering the overall context, it would be more realistic to translate it as “objective judgment,” so that the meaning of this sentence can be more accurately translated and conveyed. The overall point is that business English contains a large number of words that are used in multiple ways, far more complex than ordinary English, reflecting its multidisciplinary character. Instructors are required to pay attention to the distinction when tutoring business English and teach students to choose the exact meaning of words.
- Adopting the repetition method of translation: Business English is mostly used by workers in the foreign trade industry, and as China is a major trading country, the number of people using business English is naturally very large. Therefore, educators need to pay extra attention to the instruction of the skills related to business English when translating between Chinese and English. The first thing is to understand the differences between Chinese and English. Chinese often has repetitive words, reflecting the rhythm of Chinese, while English is relatively more concise and clear, focusing on the transmission of the meaning. Therefore, students can be instructed to use the repetition method when translating business English, that is, certain words are repeatedly reflected in the sentence, so as to conform to the expression effect of emphasizing a certain meaning or action in Chinese. For example, during COVID-19, import drivers were required to issue nucleic acid certificates, green travel codes, and freight information. This sentence repeats the translation of the verb “requires,” reflecting the strict control of import and export truck drivers during the New Crown epidemic.
- Adopt the translation of positive and negative words: Chinese and English expression habits are different, and there are differences between Chinese and English expressions when expressing negative concepts. For example, if “are not agreed” is translated literally as “are not agreed,” it is very awkward to read and does not conform to Chinese expression habits. The translator may choose to treat it as an affirmative translation “is against.” This kind of translation treatment is called the antithetical translation method, also known as the positive-speaking and negative-speaking translation method. The translation between prospeech and antispeech is a kind of statement conversion. Its basic mechanism of action is the difference of bilingualism in the perspective, emphasis, point of view, and feature selection or copying method in concept naming, topic formulation, mood expression, and emphasis distribution. For example, the English phrase “self-service bookstand” is in the positive form, which focuses on the subjective behavior process, while the Chinese phrase “no one sells books at the bookstore” is in the negative form, which focuses on the description of the objective status quo. The use of antithetical translation is more common in the translation of business English texts. For example, the government should not hesitate to intervene in the currency market through bold yen-selling and dollar-buying operations. The direct translation of “should not hesitate” as “should promptly” belongs to the opposite translation, which is in line with the Chinese expression habits.

The abovementioned three translation strategies are chosen for the sole purpose of pursuing the equivalence of the meaning of the source language and the target language, which coincides with the viewpoint of the language equivalence translation strategy. The language equivalence translation strategy emphasizes the reciprocity of meaning in the context, with a view to helping the continuous development of China's foreign trade.

## Figures and Tables

**Figure 1:** Number of international business English exams and growth rate in China from 2015 to 2020.

**Figure 2:** Differences between business English and general English.

**Figure 3:** Main characteristics of business English translation.

**Figure 4:** Evaluation criteria of business English translation features.

**Figure 5:** Distribution of the respondents' English proficiency level.

**Figure 6:** Descriptive statistical analysis of variables with the good translation effect.

**Figure 7:** Descriptive statistical analysis of variables with the poor translation effect.

**Figure 8:** Descriptive statistical analysis of the common variables of good and bad translation results.

**Table 1:** Correlation test results.

	*y*	*X*1	*X*2	*X*3	*X*4
*y*	1				
*X*1	0.023	1			
*X*2	0.032	−0.021	1		
*X*3	−0.014	0.015	0.024	1	
*X*4	0.018	0.036	0.025	−0.021	1

## Data Availability

The dataset is available upon request.

## References

[1] Ren Y. (2022). Thinking on English translation teaching mode in colleges and universities under network environment. *International Journal of Education and Teaching Research*.

[2] Chen J. (2022). An exploration of college English translation teaching based on situational cognition theory. *International Journal of Higher Education Teaching Theory*.

[3] Teng J., Yuan T., Qian Yu (2022). Research on innovation and development of online teaching model of Japanese translation in special period. *International Journal of Higher Education Teaching Theory*.

[4] Liang Y., Guo J., Yu H. (2022). Research on the reform strategy of college English translation teaching based on POA theory. *International Journal of Educational Management*.

[5] Chen S. (2022). The current situation and reflections on the teaching mode of translation course for business English majors in general universities. *Education Journal*.

[6] Zhang S., Fan H., Ma Y. (2022). Strategic innovation of college English translation teaching model for the new-era liberal arts education. *Education Journal*.

[7] Yang Li (2022). Exploring the effectiveness of translation teaching in college English from the perspective of chunks. *Journal of International Education and Development*.

[8] Shakina R. (2022). Our country has gained independence, but we haven’t”: collaborative translanguaging to decolonize English language teaching. *Annual Review of Applied Linguistics*.

[9] Wang G. (2022). Formative assessment system of VR teaching in English translation class. *OALib*.

[10] Li Y. (2022). On teaching English translations in colleges and universities. *Advances in Educational Technology and Psychology*.

[11] Grabowski Ł. (2022). Provoke or encourage improvements? On semantic prosody in English-to-Polish translation. *Perspectives*.

[12] Su W. (2021). How to use modern teaching methods to improve English Chinese translation ability. *OALib*.

[13] Guo Y. (2021). The introduction of reverse thinking in college English translation rducation. *Advances in Educational Technology and Psychology*.

[14] Liu S. (2021). Analysis of business English translation teaching from the perspective of the belt and road initiative. *Research on Literary and Art Development*.

[15] Wu J., Zeng Ya (2021). Application of functionalist translation theory in the teaching of business English translation. *International Journal of Educational Management*.

[16] Guo X. (2020). A probe into the cultivation of undergraduates’ cross-cultural communication awareness in the business English translation teaching at colleges. *International Journal of Education and Economics*.

[17] Jing L. I. (2019). The application of CAT tools in business English translation teaching. *JOURNAL OF INTERNATIONAL EDUCATION AND DEVELOPMENT*.

[18] Li Z. (2019). The construction of the turning classroom of business English translation teaching in higher vocational education under the internet + environment. *Frontiers in Educational Research*.

[19] Ying J. (2019). Critical thinking oriented teaching reform of business English translation. *Studies in Literature and Language*.

[20] Zhou P. (2019). Comparative study of traditional teaching method and ISAS teaching method in business English translation teaching in colleges and universities. *Frontiers in Educational Research*.

